# BID-Net: An Automated System for Bone Invasion Detection Occurring at Stage T4 in Oral Squamous Carcinoma Using Deep Learning

This article has been retracted.

**DOI:** 10.1155/2022/4357088

**Published:** 2022-01-30

**Authors:** Pinky Agarwal, Anju Yadav, Pratistha Mathur, Vipin Pal, Amitabha Chakrabarty

**Affiliations:** ^1^SCIT, Manipal University Jaipur, India; ^2^Department of Computer Science and Engineering, National Institute of Technology Meghalaya, Shillong, India; ^3^Department of Computer Science and Engineering, Brac University, Dhaka, Bangladesh

## Abstract

Detection of the presence and absence of bone invasion by the tumor in oral squamous cell carcinoma (OSCC) patients is very significant for their treatment planning and surgical resection. For bone invasion detection, CT scan imaging is the preferred choice of radiologists because of its high sensitivity and specificity. In the present work, deep learning algorithm based model, *BID-Net*, has been proposed for the automation of bone invasion detection. *BID-Net* performs the binary classification of CT scan images as the images with bone invasion and images without bone invasion. The proposed *BID-Net* model has achieved an outstanding accuracy of 93.62%. The model is also compared with six Transfer Learning models like VGG16, VGG19, ResNet-50, MobileNetV2, DenseNet-121, ResNet-101 and BID-Net outperformed over the other models. As there exists no previous studies on bone invasion detection using Deep Learning models, so the results of the proposed model have been validated from the experts of practitioner radiologists, S.M.S. hospital, Jaipur, India.

## 1. Introduction

Oral cancer is the sixth most dangerous cancer among all types of cancers worldwide [1]. India reports the highest number of oral cancer cases and it accounts for one-third of the total number of cases globally. There are 77,000 new cases and 58,000 mortalities turn up every year in India which is almost one-fourth of the global cases [2]. The prime contributors for oral cancer include excessive use of alcohol, tobaccos like cigarettes, chewing of betel nut, and human papillomavirus (HPV). The increasing numbers of oral cancer cases are causing great concern among Indian health communities as they are discovered only after they have reached the advanced stages. In India, 70% of the oral cancer cases are detected in the advanced stage and due to this late detection survival rate is very less [3]. Generally, oral squamous cell carcinoma (OSCC) tumors are detected in the advanced stage because these tumors do not show clinical symptoms at earlier stages. Therefore, these clinical examinations have to be supplemented with radiological imaging techniques to calculate accurate tumor size, depth of invasion and bone invasion(BI), etc. Various imaging techniques are used in oral cancer treatment. Suitable use of imaging techniques helps to understand staging of malignancy spread of the tumor to lymph nodes(LN) or distant organs and examination of vascularity. Additionally, imaging helps in the planning of resection, TNM staging, and their treatment.

The TNM staging system is introduced by the American Joint Committee on *Cancer*/Union for International *Cancer* Control and is a widely accepted staging system for cancer stage calculation.  Table 1 represents the 8th edition of the TNM stage classification given by AJCC. TNM staging framework helps to improve outcome prediction, decision making, and future research. As the name suggests, it has 3 main parts: Tumor(T), Node(N), Metastasis(M). Work of this paper focuses on the tumor part of TNM staging because bone involvement takes place in the T4 stage. From Table 1, it is clear that the tumor part is further classified and assigned a number (0–4) based on the size of the tumor and invasion of the tumor in nearby areas like cortical bones, masticator space, maxillary sinus, skull base, etc.

In 1977, the first manual for TNM staging was published by AJCC and since then bone invasion is considered the most important factor for T4 staging. There exists a significant relationship between bone involvement and chances of distant metastasis and treatment failure [5]. Detection of bone invasion in OSCC is not only essential from the tumor staging point of view but also for treatment planning and surgical resection [3]. Therefore, an underestimation of bone involvement may lead to locoregional recurrence and distant metastasis whereas overestimation of this can lead to unnecessary resection and treatment. In 12%–88% cases, OSCC tumors destruct surrounding bone areas. Clinical inspection of OSCC patients which embraces direct examination and palpation plays a key role in the detection of bone involvement [6]. But, the above-mentioned points raised a need for an accurate imaging method that can help to detect bone invasion in OSCC patients. Various imaging methods exist for the detection of bone invasion like computed tomography (CT) scan, Magnetic resonance imaging (MRI) scan, X-ray, positron emission tomography (PET) scan, bone scanning, and ultrasonography (USG). Each modality has its benefits and limitations. However, the results given by the CT scan technique in the examination of cancerous tumors are quite significant because radiologists can see both soft tissue and bone involvement in the same test. It also has high specificity (87%) and high sensitivity (96%) for bone erosion detection [7, 8].

But, the detection of bone involvement in CT images is a challenging task as image classification because a subtle erosion of the bone by the tumour is difficult to interpret by the naked eyes of radiologists. Early detection of bone involvement in CT-images followed by the proper treatment can reduce the risk of deaths and unnecessary biopsies.

To address the issue of early detection of bone invasion, work of this paper portrays a fully automated system BID-Net that aims to perform early detection of bone invasion in CT images. As an artificial neural network (ANN) model is good at classifying the images but it cannot handle the complex medical images with pixel dependencies therefore Convolution Neural Network(CNN) model has been incorporated in the proposed model as it avoids the manual feature extraction and also uses local connections and weight sharing. In the proposed model *BID-Net*, pooling layer performs down sampling thereby reducing the number of parameters and computational cost. At the same time, it is highly invariant for spatial and temporal dependencies. The prime contributions of the work has been summarised as follows:

1. Collection of CT images from S.M.S. Hospital, Jaipur to generate the dataset as there is no publicly available dataset.
2. *BID-Net* model is proposed to automate the bone invasion detection in early stage.
3. Rigorous hyper tuning of various parameters of proposed *BID-Net* model.
4. Performance analysis and comparison of proposed *BID-Net* with other benchmark and standard CNN based models i.e., Transfer learning (TL) models like VGG16 [9], VGG19 [9], ResNet-50 [10], MobileNet V2 [11], DenseNet-121 [12], and ResNet-101 [10].

The simulation results affirm that the proposed *BID-Net* outperforms the other simulated benchmark CNN based architectures. The rest of the paper is organized as follows: Section 2 presents the literature survey.  Section 3 describes the dataset and methodology that drives the proposed *BID-Net*.  Section 4 shows comparative analysis of the proposed *BID-Net* model with other simulated TL models.  Section 5 concludes the paper and outlines the scope for future research.

## 2. Literature Survey

In this section a detailed related work is discussed. DL techniques have revolutionized the medical imaging areas like radiology, digital whole slide imaging, etc. Literature survey is classified into three parts. Firstly, the papers concerning benign and malign classification of oral cancer are discussed. Next, papers regarding stage classification of oral cancer are added. After that, papers on bone metastasis and bone invasion are included.Welikala et al. presented a multi-class image classification and detection model for oral lesion detection and classification. They used ResNet101 for classification and faster R–CNN for detection with F1-score attained as 41.31% and 33.03% respectively [13]. Fu et al. proposed a cascade CNN-based model on OSCC photographic image dataset. The detection model takes the OSCC image as input and creates a bounding box around the suspected lesion area. That particular lesion area is cropped as fed to the classification model for binary classification. The results attained by them were within 95% of CIs. Some authors used hyperspectral images for oral cancer detection [14]. Ijaz et al.developed a classification model which takes risk factors as input. The authors used density-based spatial clustering of applications with noise (DBSCAN) and isolation forest (iForest) as pre-processing technique for outlier detection and Random Forest is used as a classifier [15]. Mandal et al. formed an ensemble by using four filter methods for disease prediction and features from the ensemble are accessed by the three classification models [16].

CT and MRI images also have a significant impact on oral cancer detection. In 2018, Huang et al. developed a DCNN model for automatic GTV contouring on PET-CT images of 22 head and neck cancer (HNC) patients [17]. In 2019, Xu et al. compared 2DCNN and 3DCNN models to classify benign and malign oral cancer tumors on CT scan images of OSCC patients [18]. Ma et al.proposed a DL model to classify cancerous and non-cancerous tissue in an animal model using hyperspectral images. An autoencoder is used to reclassify the misclassified pixels by using the adaptive weights and then the autoencoder is retrained on these updated pixels. The sensitivity and the specificity achieved by the model was of 92.32% and 91.31% respectively [19]. I 2020, Kawauchi et al. proposed A CNN model which is based on residual network(ResNet) on Pet-CT images of 3485 patients. The results of CNN are classified into 3 categories and are generated on the patient level and regional level. The classification accuracy for benign, malign, and equivocal classes is attained as 99.4%, 99.4%, and 87.5% respectively whereas the accuracy of region-based analysis for head and neck, chest, and abdomen region is achieved as 97.3%, 96.6%, 92.8%, and 99.6%, respectively [20].Ren et al. utilize machine learning technique on MRI images of 80 patients to classify these images in well-differentiated and moderately or poorly differentiated categories. For this, 1118 features were extracted, reduced using reproducibility analysis, selected using minimum-redundancy maximum-relevance algorithm (MRMR), and the model is classified using 3 different classifiers and Random forest performed best with receiver operating characteristic curve(ROC) curve as 93.6 and accuracy as 86.3% [21]. Rahman et al. presented an ML model for classification in the normal and malignant cells on histopathological images using supper vector machine classifier [22]. Aubreville et al. worked on CLE images to differentiate between malignant and non-malignant tumors with 88.3%accuracy [23].In 2019, Halicek et al. used four dissimilar models for lesion segmentation on WSI images. They tried to generalize their results a test dataset from the different cohorts [24]. Du et al. utilized Multilayer perceptron and Gaussian Mixture Model (GMM) classifiers on the dataset of 75 patients to perform a comparative analysis of classification accuracy of the TNM staging system [25]. Rajaguru proposed a model based on machine learning(ML) techniques to classify MRI datasets in two groups stage I-II AUCs of 0.853 and 0.849 respectively [26]. In 2018, Kann et al. deployed a 3 DCNN model for identification of lymph nodes and extra-nodal extension in 2,875 CT image datasets. the model has predicted the Are under curve (AUC) value as 91% [27].Chen et al. combined ML and DL techniques to make a hybrid model that can gain advantages of both hand-crafted features and automated generated features to predict lymph node metastasis in HNC patients. The authors have performed multi-class classification by categorizing the dataset into three categories: normal, suspicious, and having LNs. Comparative analysis was performed among hybrid model, XmasNet, and Radiomics model and these models achieved accuracy as 0.88, 0.81, and 0.75 on PET images respectively [28]. In 2021, Ariji et al. presented a DetectNet model to detect cervical LN metastasis, with 90% accuracy, on 365 CT scan images of OSCC patients [29].

Bone metastasis (BM) is bit different from BI. BI is the condition where tumour cells expand into nearby bones whereas BM is the condition where primary tumour spreads to the new location, forms secondary tumour and spreads to the bones. Breast, prostate, and lung cancer are the most common cancer affected by BM.Papandrianos et al. proposed a CNN model and compared it with popular TL models like VGG 16, ResNet-50, MobileNet, and DenseNet, to classify bone scintigraphy images of breast cancer patients. They classified images into two categories: bone metastasis and non- metastasis with an accuracy of 92.50% [30]. A similar kind of work is performed by the same authors in prostate cancer [31]. Zhao et al.proposed a DL model where the same model architecture is used to classify BM condition in Breast *Cancer*, Prostate *Cancer*, Lung *Cancer*, and other cancers also. The resulted ROC for Breast *Cancer* was 98.8%, Prostate cancer 95.5%, Lung cancer 95.7%, and other cancers 97.1% [32].Some researchers [33–35] have worked on the problem of bone loss which is not related to oral cancer. But the causes of boss loss in these papers are Rheumatoid Arthritis (RA), Periodontitis, and Musculoskeletal conditions. From literature it has been observed that there exists no research paper dealing with the problem of bone invasion in OSCC patients using ML and DL techniques.

## 3. Data Set Description and Proposed Methodology

### 3.1. Data Description

The dataset collection for this work is collected from Sawai Man Singh (SMS) Hospital, Jaipur, India. Total 1755 CT scan images of 36 patients have been retrospectively collected from July 15th, 2020 to April 30th, 2021.  Figure 1 represents sample images. Figures 1(a)–1(c) demonstrate the images with bone invasion while Figures 1(e)–1(g) shows the cases without bone invasion. There is a significant difference in the gender of patients. There were 32(89%) male and 4(11%) female patients in the dataset of 36 patients with a mean age of 43.95 years. Out of 1755 images, 915 CT images showed bone invasion in 19 patients whereas 840 images of 17 patients were without bone invasion. Most of the cases having bone invasion were in the advanced stage. Out of 19 patients of bone invasion, 15 (79%) were in the clinical T3 stage and 4(21%) cases were in the T4 stage. There was no case of the T1 and T2 stages. Cases where CT images showed bone loss due to other reasons like age factor, fracturing, Rheumatoid arthritis, and chronic kidney disease, etc are excluded. All CT images are histologically proven and classified in the respective groups accordingly.

Philips ingenuity 128 slice CT scanner machine is used for CT examination. Patients were injected with IOHEXOL 300 mg to get contrast-enhanced CT images. Slice thickness and the interval between slices were 1.55 mm and 0.75 mm respectively. All images have been acquired in dicom format with a resolution of 1183 × 1067 pixels in an axial plane. Following Table 2 shows the percentage of OSCC patients at different locations in the oral cavity. Among all the collected images, 4 (21%) were of Ca-tongue, 14(74%) Ca-buccal mucosa, and 1(5%) Ca-lip of the oral cavity.

### 3.2. Proposed Methodology and Architecture of BID-Net

In this section proposed methodology, architecture of *BID-Net* model and quantitative analysis parameters are discussed in detail.

#### 3.2.1. Proposed Methodology

Figure 2 demonstrates the working diagram of the proposed architecture for BI detection from the CT images. It is divided into 5 sections: Data acquisition, Image Pre-processing, Train-Test split, comparison with TL and Results. Details of each section is given below.

 
*Data Acquisition* The proposed *BID-Net* model targets OSCC patients. As no public dataset is available to develop the proposed model, therefore, CT images of oral patients have been collected and annotated by the experienced radiologists from the S.M.S. hospital, Jaipur. Detailed dataset description has been already discussed in Section 3.1.
 
*Image Pre-processing* Generally, the image format for medical images is DICOM. These DICOM files are very bulky and take lots of computation time. Hence, the format of images has been changed from DICOM to PNG. Images are resized to 224 × 224 × 3 and then data augmentation techniques like horizontal flip, vertical flip shear and zoom are used to increase the size of train dataset. Images were normalized using min-max normalization technique and rescaled within the range of 0 to 1.
 
*Train–test split* The proposed *BID-Net* architecture has been trained on 80% training dataset and is tested on 20% of the total dataset. This particular division is chosen because the size of training dataset has been increased by augmentation technique.
 
*Transfer Learning Models* A requirement of the computational power and a large dataset is the biggest issue faced by the researchers. TL models handle these problems very efficiently as these models are trained on a large number of datasets such as ImageNet and the features extracted by these models can be transferred to the other same type of problem. Researcher are facing the scarcity of the massive image dataset in the medical field TL models came out as a wonderful option to solve the problem of dataset shortage. When TL models are used as feature extractor, all the layers of pre-trained models are frozen, a new classifier is added on the top and the classifier is trained from the scratch on top of the previously trained model.

#### 3.2.2. BID-Net Architecture

To propose the *BID-Net* on our dataset we had performed a rigorous experiment on different values of hyper parameters like image size, kernel size, no of kernels, dropout rate, etc have been performed. To determine the best input size, the input image is resized on three different values: 128 × 128, 224 × 224. The best results are obtained for 224 × 224. Experiments on the number of kernels at the third convolution layer has been carried for two values: 32 and 64 for kernel. 64 came out as the winning number. The dropout rate is also taken as 0.25, 0.50, and 0.70 and 0.25 made the best efforts to remove overfitting.

Figure 3 demonstrates the architecture of the proposed *BID-Net* model. Input to the model is RGB CT scan images of size 224 × 224 which has been provided by pre-processing. *BID-Net* has 3 convolution layers and each convolution layer is followed by the pooling layer. The first and second convolution layer has 32 filters while in the third layer this number has been doubled i.e., 64. The size of the kernel is kept 3 × 3 across all the layers. RELU activation function is used et al.l the layers. Filters used et al.l the pooling layers are the size of 2 × 2. Image size after the third pooling layer is reduced to 26 × 26 × 64 and flattened for fully connected layers. Next, the output generated by the flattened layer i.e., one-dimensional array is given as input to the dense layer having 64 neurons. Finally, there is an output layer with a softmax activation function for binary classification. Adam optimizer has been employed. Batch size and learning rate are set as 32 and 0.000 1 respectively.  Table 3 illustrates the various parameters of the proposed *BID-Net* model architecture.

Six popular TL models VGG16, VGG19, ResNet-50,DenseNet-121, ResNet-101 and MobileNet V2 are used as feature extractors for performance comparison with the proposed BID-Net.

### 3.3. Evaluation Metrics

The model is trained on 80% of the training dataset and 20% of the test dataset. The performance of the simulated models is evaluated and compared on accuracy, F1-score, precision, and recall as given in equations (1)–(4) respectively. For the given value of TP(BI, BI) = (True positive: the image label is BI and it is correctly classified.), TN(NBI, NBI) = (True negative: the label on the image is no BI and is correctly classified.), FP(NBI, BI) = (False positive: the image label is no BI and the image is wrongly classified as BI), FN(BI, NBI) = (False negative: the label on images is BI and the image is wrongly classified as no BI). The performance metrics have been calculated as:

(1) $$\begin{array}{c} \text{Accuracy}=\frac{TN_{\text{INB},\text{INB}}+TP_{BI,BI}}{TP_{BI,BI}+FP_{\text{NBI},BI}+TN_{\text{INB},\text{INB}}+FN_{BI,\text{NBI}}}\times 100, \end{array}$$

(2) $$\begin{array}{c} \text{Precision}=\frac{TP_{BI,BI}}{TP_{BI,BI}+FP_{\text{NBI},BI}}\times 100, \end{array}$$

(3) $$\begin{array}{c} \text{Recall}=\frac{TP_{BI,BI}}{TP_{BI,BI}+FN_{BI,\text{NBI}}}*100, \end{array}$$

(4) $$\begin{array}{c} F1-\text{score}=2*\frac{\text{Recall}*\text{precision}}{\text{Recall}+\text{Precision}}*100. \end{array}$$

#### 3.3.1. Kappa Coefficient

Kappa coefficient is an important performance metric for imbalanced data set. As the data set in the proposed work is slightly imbalanced, Kappa coefficient for all the models is also calculated. It measures the agreement between ground truth labels and the labels predicted by the classifier. It compares observed accuracy with expected accuracy. Equation (5) is used to calculate kappa coefficient.

(5) $$\begin{array}{c} \text{Kappa}-\text{coefficient}\left(k\right)=\frac{\left(P_{0}-P_{e}\right)}{\left(1-P_{e}\right)}. \end{array}$$

Here, Po and Pe represent the observed accuracy and expected accuracy.Value for the Kappa coefficient is between 0 and 1. A zero denoted no agreement and one denotes perfect agreement. According to Fleis, kappas greater than 0.75 are excellent, kappas between 0.40 and 0.75 are fair to good, and less than 0.40 are considered poor [36].  Table 4 represents kappa values for all the classifiers. Kappa coefficient for *BID-Net* is 0.79 and close to perfect classification and it is highest among all the classifiers. Kappa values for other classifiers lies between 0.2 and 0.5.

ROC Curve The ROC is used to plot the true positive rate against the False positive rate at different threshold values. AUC curve differentiates between two classes. ROC curve gives best prediction results at point (0,1) of ROC space. This point is called perfect classification and represents 100% specificity (no false positive) and 100% sensitive (no false negative).

## 4. Result Analysis

This section describes the experimental setup and performance evaluation of BID-Net and compares the performance of *BID-Net* with the other standard TL models.

### 4.1. Experimental Setup

Google collaborator (Google collab) is used to train and evaluate the models.The motive to use Google collab is that it provides free GPU. Keras 2.4.3 package, TensorFlow 2.4.1, and python 3.7 are used for model implementation. For the optimization process, Adam optimizer is preferred and each model is run for 50 epochs. For TL models, ImageNet weights are used for weight initialization in all the pre-trained models thereby avoiding random weight initialization. As the dataset is small in size TL models are used as feature extractor. In this case, all the layers of pre-trained models are frozen, a new classifier is added on the top and the classifier is trained from the scratch on top of the previously trained model. For TL models also images were resized to 224 × 224. Detailed architecture diagram of VGG-16, VGG-19, ResNet-50, and MobileNetV2 can be seen in Figure 2.

### 4.2. Performance Result Analysis

The dataset is divided into training and testing sets. The 80% portion of total dataset is for training and 20% for testing.  Figure 4 demonstrates the learning curves for *BID-Net* where Figure 4(a) shows the loss curve and Figure 4(b) depicts the accuracy curve. Figure 4(a) shows that BID-Net gives minimum loss at epoch 28 and after that there is not significant decrease in the loss is observed. Figure 4(b) demonstrates that the accuracy of the model sharply goes up on executing the model from epoch 0 to 50. On 28th epoch, model attained the highest accuracy and after that there is a random increase and decrease in the accuracy. This random change in accuracy proves that model learned dataset and parameters gradually.

To fine tune the hyperparameters, proposed model *BID-Net* and other model have been trained on four learning values: 0.01, 0.001, 0.001 and 0.000 1.  Table 5 below shows the effect of learning rate on the various performance matrices of each model. *BID-Net* has achieved highest accuracy, F1-score, precision and recall value at 0.000 1 learning rate. The highest accuracy, F1-score, Precision and recall of 93.62, 92.63, 91.00 and 95.17 respectively has been achieved by the proposed *BID-Net* while the lowest accuracy, F1-score, Precision and recall of 80.40, 77.02, 75.54 and 81.90 has been attained by ResNet-101. This is because ResNet-101is a complex model and needs large amount of training dataset to give accurate results.

Confusion matrix is shown in Figure 5. From the confusion matrix, it is clear that miss-classification for positive class (bone invasion) is 2.01% and for negative class (No Bone Invasion) is 7.38%. Hence, the results achieved by our model are very significant when compared with other models.

*BID-Net* is compared with six popular TL models: VGG-16, VGG-19, ResNet-50, DenseNet-121,Res Net-101 and MobileNetV2 on the same dataset.  Figure 6 demonstrates the comparison of *BID-Net* with VGG-16, VGG-19, ResNet-50, DenseNet -121, ResNet-101 and MobileNetV2 in terms of accuracy. From Figure 6, it is clearly seen that *BID-Net* has attained the highest accuracy of 93.62% whereas the lowest accuracy 82.92% is given by ResNet-101.

The ROC curve for multiple classifiers is shown in Figure 7. ROC curve for *BID-Net* is almost near to (0, 1) that signifies that the classification done by *BID-Net* is near to perfect classification. The graph clearly states that the highest AUC score is attained by *BID-Net* see Figure 7.

### 4.3. Execution Time Analysis

In medical imaging, the execution time of the models plays a key role. All the models have been compared in terms of execution time.  Figure 8 demonstrates the comparative analysis of all the models in terms of time. Execution time for ResNet-101 is highest (90 min) whereas *BID-Net* took the lowest execution time (30 min). This is because ResNet-101 architecture is very complex and involves a higher number of trainable and non -trainable parameters. Total number of parameters for ResNet-101 is 42,858,882 whereas *BIT-Net* model is optimized so it has a lesser number of parameters. Total number of parameters for *BIT-Net* is 2,797,730 This depicts the computational complexity of the models. It means, if a technique takes more memory space, it takes longer time to execute.

To our best knowledge, we did not find any work on BI classification using deep learning. Therefore it became essential to validate the model from experts. The model was validated by practitioner radiologist of hospital. The results were found very satisfactory by radiologist.

## 5. Conclusion

DL techniques are getting a lot of popularity and attention in the medical imaging field. DL techniques provide accurate and cost-effective solutions. The work of this paper presented a DL based framework, named *BID-Net*, that is a system for bone invasion detection in Oral Squamous carcinoma. In the presented work, CT- scan images of oral cancer patients are collected from SMS Hospital, Jaipur, India. The generated dataset was labelled with the help of experts. Various CNN parameters are experimented to get the best configured CNN model. Performance of the proposed *BID-Net* model is also compared with six standard TL models. The simulation results confirmed that the proposed BID-Net has achieved outstanding accuracy and is cost-effective as well. *BID-Net* model can classify CT images of OSCC patients with 93.62% accuracy within minimal time. The loss generated by the proposed model *BID-Net* model is also very low. Miss-classification in both positive and negative classes is very less. For positive class (images with bone invasion), miss-classification is 2.01% whereas for negative class (images without bone invasion), it is only 7.38%. The Auc value for our model is 95.9% and this value is also very high which shows the performance of our model is quite good. Detection of bone invasion in OSCC is not only essential from the tumor staging point of view but also for treatment planning and surgical resection. Therefore, timely detection of bone involvement is very important because underestimation of bone involvement may lead to locoregional recurrence and distant metastasis whereas overestimation of this can lead to unnecessary resection and treatment. As this work is the first of its kind for the detection of bone involvement in CT images, results of the proposed model have also been validated from professional experts. The dataset does not have the cases of bone loss due to other factors like age factor, fracturing, Rheumatoid arthritis, and chronic kidney disease, etc. The size of the dataset is also limiting the present work. For future work, these cases can also be considered.

## Figures and Tables

**Figure 1:** Image samples of OSCC patients (Labels: (a, b, c) with BI, (d, e, f) without BI.

**Figure 2:** Block diagram of the proposed Methodology of *BID-Net* model.

**Figure 3:** Architecture of *BID-Net* for BI classification.

**Figure 4:** Learning curves for *“BID-Net”*: (a) loss curve (b) accuracy curve.

**Figure 5:** Confusion matrix of the proposed *BID-Net* model.

**Figure 6:** Comparative analysis of proposed model *BID-Net* and TL models in terms of accuracy.

**Figure 7:** ROC curve of all models in a single plot.

**Figure 8:** Comparison of proposed model *BID-Net* with other TL models in respect to time.

**Table 1:** Eighth edition of *T* stage classification given by AJCC for oral cancer [4].

P	Primary tumor of the oral cavity
Tx	Primary tumor cannot be accessed.
Tis	Carcinoma in situ
T1	Primary tumor has a maximal diameter of 2 cm
T2	Primary tumor has a maximal diameter of more than 2 cm but no more 4 cm
T3	Primary tumor has a maximal diameter of more than 4 cm.
T4a (oral cavity)	Tumor invades through cortical bone, into deep/extrinsic muscle of tongue, maxillary sinus, or skin of face
T4b	Tumor invades masticator space, pterygoid plates, or skull base; or encases internal carotid artery

**Table 2:** Percentage of OSCC patients at different locations in the oral cavity of BI patients.

Cancer type	Patients in(%)
Ca-buccal mucosa	14 (74%)
Ca-tongue	4 (21%)
Ca-lip	1 (5%)
Total no. patients	19

**Table 3:** Hyper tune parameters of *BID-Net* for BI.

Type of layer	Size	Channel	Filter size	Activation function	No. of parameters
Convo1	222 × 222 × 32	32	3 × 3	Relu	896
Pool1	111 × 111 × 32	—	2 × 2	—	0
Convo2	109, 109, 32	32	3 × 3	Relu	9248
Pool2	54 × 54 × 32	—	2 × 2	—	0
Convo3	52 × 52 × 64	64	3 × 3	Relu	18 496
Pool3	26 × 26 × 64	–	2 × 2	–	0
Flatten	43 264	–	—	—	0
Dense 1	64	–	—	—	2768 960
Dropout	64				0
Dense 2	2	–	–	–	130

**Table 4:** Kappa coefficient of different models.

Models	Kappa-coefficients
BidNet	0.79
ResNet-101	0.54
DenseNet-121	0.51
ResNet-50	0.49
Vgg-19	0.49
MobileNetV2	0.375
Vgg-16	0.22

**Table 5:** Effect of learning rate on model's performance.

Learning models	Learning rate	Accuracy	F1-score	Precision	Recall	AUC-score
BID-net	0.01	90.6	89.12	87.68	91.32	94.58
	0.001	91.27	90.16	88.39	93.86	93.24
	**0.000 1**	**93.62**	**92.63**	**91**	**95.17**	**95.9**
	0.000 01	80.2	72.85	77.77	70.88	93.37
VGG-16	**0.01**	**87.87**	**84.62**	**85.33**	**83.39**	**86.7**
	0.001	85.95	82.12	82.9	81.44	87.29
	0.000 1	83.19	78.33	79.51	77.4	84.42
VGG-19	0.000 01	70.79	57.88	60.86	57.56	72.04
	0.01	84.47	79.78	79.3	80.33	86.01
	**0.001**	**84.84**	**80.46**	**81.73**	**79.46**	**85.64**
	0.000 1	78.78	70.54	74.35	68.87	83.23
	0.000 01	68.87	51.8	55.22	52.88	70.47

ResNet-50	0.01	83.47	79.66	79.33	80.03	84.82
	0.001	79.33	70.83	75.58	68.95	86.87
	0.000 1	84.29	79.88	80.86	79.08	89.95
	**0.000 01**	**85.67**	**82.27**	**82.08**	**82.47**	**90.1**
MobileNet	0.01	84.16	79.23	80.45	79	88.95
	0.001	81.54	76.35	77.22	75.65	85.59
	**0.000 1**	**82.92**	**77.43**	**79.6**	**75.99**	**89**
	0.000 01	76.3	64.89	71.1	63.5	80.64
DenseNet121	0.01	82.65	82.01	83.58	81.13	89.18
	0.001	83.98	83.61	83.31	84.18	91.37
	**0.000 1**	**84.43**	**75.3**	**83.42**	**72.1**	**94.5**
	0.000 01	78.51	78.61	78.31	79.12	90.12

ResNet101	0.01	79.25	76.37	75.32	82.69	88.9
	0.001	78.09	69.13	70.31	68.28	89.45
	0.000 1	76.08	74.18	75.17	83.17	87.21
	**0.000 01**	**80.4**	**77.02**	**75.54**	**81.9**	**88.5**

## Data Availability

The data used to support the findings of this work is available with Sawai Man Singh Hospital, Jaipur, India.
